# Toward Bioremediation of Methylmercury Using Silica Encapsulated *Escherichia coli* Harboring the *mer* Operon

**DOI:** 10.1371/journal.pone.0147036

**Published:** 2016-01-13

**Authors:** Aunica L. Kane, Basem Al-Shayeb, Patrick V. Holec, Srijay Rajan, Nicholas E. Le Mieux, Stephen C. Heinsch, Sona Psarska, Kelly G. Aukema, Casim A. Sarkar, Edward A. Nater, Jeffrey A. Gralnick

**Affiliations:** 1 BioTechnology Institute, University of Minnesota-Twin Cities, St. Paul, Minnesota, United States of America; 2 Department of Biochemistry, Molecular Biology, and Biophysics, University of Minnesota-Twin Cities, Minneapolis, Minnesota, United States of America; 3 Department of Soil, Water, and Climate, University of Minnesota-Twin Cities, St. Paul, Minnesota, United States of America; 4 Department of Biomedical Engineering, University of Minnesota-Twin Cities, Minneapolis, Minnesota, United States of America; 5 Department of Microbiology and Immunology, University of Minnesota-Twin Cities, Minneapolis, Minnesota, United States of America; University of Houston, UNITED STATES

## Abstract

Mercury is a highly toxic heavy metal and the ability of the neurotoxin methylmercury to biomagnify in the food chain is a serious concern for both public and environmental health globally. Because thousands of tons of mercury are released into the environment each year, remediation strategies are urgently needed and prompted this study. To facilitate remediation of both organic and inorganic forms of mercury, *Escherichia coli* was engineered to harbor a subset of genes (*merRTPAB*) from the mercury resistance operon. Protein products of the *mer* operon enable transport of mercury into the cell, cleavage of organic C-Hg bonds, and subsequent reduction of ionic mercury to the less toxic elemental form, Hg(0). *E*. *coli* containing *merRTPAB* was then encapsulated in silica beads resulting in a biological-based filtration material. Performing encapsulation in aerated mineral oil yielded silica beads that were smooth, spherical, and similar in diameter. Following encapsulation, *E*. *coli* containing *merRTPAB* retained the ability to degrade methylmercury and performed similarly to non-encapsulated cells. Due to the versatility of both the engineered mercury resistant strain and silica bead technology, this study provides a strong foundation for use of the resulting biological-based filtration material for methylmercury remediation.

## Introduction

Microbial transformation of metals has a large impact on biogeochemical cycles and can alter metal distribution and partitioning in the environment. Alterations, such as change in redox state and conversion between organic and inorganic states, affect solubility and toxicity of metals and hence have great impact on environmental and public health [1,2]. Toxicity of the metal mercury is a particular concern at present because mono-methylmercury (hereafter, methylmercury), the most common organic form, is a neurotoxin that biomagnifies in the food chain [3]. Five thousand to 8000 tons of mercury are estimated to be emitted into the atmosphere yearly from both human and natural sources, and anthropogenic emissions are expected to increase through 2050 [4]. Current remediation strategies exist for mercury but are prohibitively costly in many environments and other solutions are needed [5].

Bioremediation offers a potentially cost-effective and environmentally conscious approach to the problem of mercury pollution. An attractive biological-based remediation strategy for mercury pollution is utilization of the *me*rcury *r*esistance (*mer*) operon found in bacteria. The *mer* operon exists in a variety of structures and organizational forms, and a few key genes have become the central targets for remediation efforts [5]. Essential to remediation of both organic and inorganic forms of mercury are the key enzymes MerB and MerA, respectively. MerB cleaves the C-Hg bond of organomercurials through protonolysis resulting in Hg(II) that is then reduced by MerA, the mercuric reductase, to volatile Hg(0) [2, 6]. Other genes important to the system include *merP* and *merT* that encode for an Hg(II) transport system across the periplasm and inner membrane, and *merR* that encodes for the mercury-specific regulator of the operon [2, 7].

Previous bioremediation approaches for mercury have centered on usage of bacteria with engineered or naturally occurring *mer* operons and/or a variety of metal binding proteins. Genetic engineering has been used to introduce parts from the *mer* operon into a variety of hosts proposed for use in mercury removal from contaminated sites [8–10]. Other studies have focused on engineering bio-sorbent strains utilizing Mer proteins and/or metal binding proteins or chelators such as metallothionein and polyphosphate kinase [11–19]. Bio-sorbent strains are limited by their metal retention capacity, and because sorption is a passive process, strains must be regenerated after reaching saturation. Use of bio-sorbent strains also requires methods to separate mercury from biomass for recovery. The only method to date able to recover mercury and work at technical scale is the use of natural *mer*-containing strains of *Pseudomonas* adsorbed to silica pumice granules in packed bed bioreactors [20, 21]. Because adsorbed cells can easily be released in effluent water, engineered strains cannot be used with this type of system [20]. Also, the formation of biofilm and exopolysaccharide within pumice material may limit diffusion in flow-through systems. Here we describe the use of a silica gel whole cell encapsulation system to address these challenges.

Silica encapsulation has previously been used in atrazine bioremediation [22, 23], providing protection of the biocatalyst, avoidance of dispersal of organisms, and overall mechanical structure that broadens possible engineering applications. Silica gels are formed by condensation or gelation of a hydrolyzed silicon alkoxide crosslinker into a solid silica matrix. Following cross-linker hydrolysis, cells added during condensation become entrapped within the gel matrix [22]. Recent improvements in encapsulation technology have resulted in methods retaining cell viability, which is imperative for mercury remediation since reduction of Hg(II) by MerA is an NADPH-dependent reaction [2, 23]. Encapsulated cells have been shown to retain high enzymatic activity over a period of months [23]. Optimization and modeling studies are also available to minimize material cost and pressure drop in packed beds while maintaining material strength [24].

## Materials and Methods

### Bacterial Strains and Culture Conditions

*E*. *coli* strain MG1655 was kindly provided by Dr. Arkady Khodursky (University of Minnesota). *E*. *coli* strains UQ950 and WM3064 used for cloning and conjugal transfer have been described previously [25]. For routine propagation of *E*. *coli*, single colonies from freshly streaked -80°C stocks were used to inoculate cultures grown for 16 hours in Luria Broth (LB) medium supplemented with 50 μg mL^-1^ kanamycin when appropriate. Unless specified otherwise, cultures were grown in LB, shaken continuously at 250 rpm, and incubated at 37°C.

### Reagents and Materials

Enzymes were purchased from New England Biolabs (Ipswich, MA). Kits for gel purification and plasmid mini preps were purchased from Qiagen (Valencia, CA). All related reactions were carried out according to manufacturer instructions.

Media components, including Noble agar, were purchased from Becton, Dickinson and Company (Sparks, MD). Chemicals for encapsulation including Ludox TM40, alkoxide tetramethyl orthosilicate (TMOS), and Polyethylene Glycol 600 were purchased Sigma-Aldrich (St. Louis, MO). Mercuric chloride and methylmercury chloride were purchased from Fisher Chemical (Pittsburgh, PA). Due to the toxicity of mercury compounds, all safety protocols and operating procedures were reviewed by the Department of Environmental Health and Safety at the University of Minnesota.

### Plasmid Construction

Plasmid pDU1358 was kindly provided by Dr. Anne Summers (University of Georgia, Athens) [26]. Plasmid pBBRBB has been described previously [27]. Genes *merRTPAB* were amplified from pDU1358 in two stages to enable incorporation in the BioBrick compatible vector pBBRBB. First, a portion of *merA* and *merB* were amplified using primers merAmut-F (GTCGCGCATGTGAACGGCGAGTTCGTGCTGACCACGGGACA) and merB-R (nnACTAGTTCACGGTGTCCTAGATGACA) to mutate the internal EcoRI restriction site (bp 1024–1029) within *merA*. The resulting fragment was then gel purified and used to prime the second reaction along with primer merR-F (nnTCTAGACTACACCGCGTCGGCACCAC) to amplify *merRTPAB*. This fragment was digested with XbaI and SpeI, gel purified, and cloned into the corresponding sites of pBBRBB generating plasmid pBBRBB::*mer*. Constructs in the pBBRBB backbone were moved into *E*. *coli* by conjugal transfer using donor strain WM3064.

### Zone of Inhibition Plate Assays

*E*. *coli* strains were picked from single colonies into LB medium supplemented with 50 μg mL^-1^ kanamycin. Overnight cultures were diluted 10-fold, and 3 mL was added to tryptone medium agar plates (containing per liter: 15 g tryptone, 5 g NaCl, 10 g Noble agar, 1 pellet sodium hydroxide). Noble agar was used to limit agar batch variability that can confound heavy metal assays. Excess culture was removed after 5 minutes, a 6 mm paper disc was added to the center of the plate, and 10 μL of a 0.1 M HgCl_2_ stock solution was added to each disc. HgCl_2_ stock solutions were made fresh for each experiment. Plates were incubated at 37°C for 16 hours after which zones of inhibition were measured as the diameter of clearing around each disc.

### Encapsulation

Methods for encapsulation were adapted from previous sol-gel techniques [23, 28] Hydrolyzed cross-linker was produced by mixing TMOS with ultrapure water and 1 M HCl (1:1:0.001 vol/vol/vol) and incubating for two hours at room temperature. A solution containing colloidal silica nanoparticles (TM40), polyethylene glycol (PEG-600) and phosphate-buffered saline (PBS) was prepared prior to encapsulation (2:2:1 vol/vol/vol). Bacteria re-suspended in PBS between 0.1–0.2 g mL^-1^ were then introduced to this solution with a 1:1 volumetric ratio to create a homogenous solution with silica interspersed between cells. Hydrolyzed cross-linker was then spiked into this solution and immediately transferred into aerated mineral oil (800 rpm, 15 min) to provide uniform viscosity throughout emulsification. After letting the silica set, beads containing the embedded bacteria were purified by phase-separation. Beads entered the dH_2_O phase of the oil-water mixture and were isolated using a separatory funnel. Samples were both washed and stored in PBS overnight at 4°C prior to methylmercury testing.

### Methylmercury Assays

Assays were conducted in acid-cleaned Balch tubes [29] containing 7 mL LB medium and 1 mg L^-1^ methylmercury chloride. Using previously published viability data for our encapsulation methods, encapsulated cells were inoculated at a cell density within an order of magnitude of that of the non-encapsulated cells [23]. For assays using encapsulated cells, 0.3 g of encapsulation material was added to each tube. For assays with non-encapsulated cells, overnight cultures were washed in minimal medium and inoculated to an initial optical density (OD_600_) of ~ 0.1. Cultures were incubated at 37°C and shaken at 250 rpm. Samples were removed for analysis at times indicated.

Samples were analyzed for monomethylmercury in the University of Minnesota Mercury Analytical Laboratory using EPA method 1630 modified to eliminate sample distillation. Samples were placed in acid-cleaned 40 mL I-chem glass vials fitted with PTFE/silicone septa and brought to a final volume of 30 mL with distilled deionized water. Samples received 0.225 mL of 2 M pH 4.5 acetate buffer and 0.03 mL of sodium tetraethylborate ethylating solution. Monomethylmercury concentrations were determined from headspace gas analysis by a Tekran model 2700 Automated MethylMercury Analyzer with Hg detection by cold vapor atomic fluorescence spectrometry (CVAFS) following capillary gas chromatography and pyrolization of ethylated Hg species.

Quality Assurance/Quality Control measures included the preparation of a calibration curve from 10 ng L^-1^ and 500 ng L^-1^ working standards at the start of each run of samples and the analysis of control check standards (0.1 and 0.5 ng L^-1^) every 10 samples. Recoveries for control check standards averaged 98%, well within acceptable values.

### Microscopy

Samples were fixed in 2% glutaraldehyde in 0.1 M sodium cacodylate buffer (pH 7.2) overnight at 4°C, rinsed in 0.1 M sodium cacodylate buffer, then placed in 1% osmium tetroxide in 0.1 M sodium cacodylate buffer overnight at 4°C. Specimens were rinsed in ultrapure water (NANOpure Infinity; Barnstead/Thermo Fisher Scientific; Waltham, Maryland), dehydrated in an ethanol series, and processed in a critical point dryer (Autosamdri-814; Tousimis; Rockville, Maryland). Material was mounted on double-sided adhesive carbon tabs on aluminum stubs, sputter-coated with gold-palladium, and observed in a scanning electron microscope (S3500N; Hitachi High Technologies America, Inc.; Schaumberg, Illinois) at an accelerating voltage of 10 kV.

## Results and Discussion

To develop a bioremediation strategy for both organic and inorganic forms of mercury, we began by cloning *merRTPAB* of the *mer* operon from pDU1358 (originally isolated from *Serratia marcescens*) into *E*. *coli* K12 resulting in strain *E*. *coli* pBBRBB::*mer* [26]. During amplification, the internal EcoRI restriction site in *merA* was mutated in order to create a *mer* cassette compatible with the biobrick cloning system and the vector pBBRBB (see Materials and Methods) [27]. Biobrick compatibility creates a plug-and-play vector system and facilitates addition of further remediation cassettes. Use of a modular approach in plasmid design allows the strain to be tailored to the specific needs of future remediation sites. Following construction, zone of inhibition plates were used to assess resistance to ionic forms of mercury by engineered strains. Strains were spread evenly on tryptone medium plates containing discs loaded with an HgCl_2_ solution. Following overnight incubation, zones of inhibition were measured as the diameter of clearing around discs (Fig 1). *E*. *coli* pBBRBB::*mer* was resistant to ionic mercury as measured zones of clearing for *E*. *coli* pBBRBB::*mer* were comparable to the positive control *E*. *coli* pDU1358 and significantly smaller (p-value = 0.0002) than control strains containing empty vector (Fig 1; Table 1).

**Fig 1:** Representative zone of inhibition from filter disc assays for mercury(II) chloride resistance for A) *E*. *coli* pDU1358 B) *E*. *coli* pBBRBB::*mer* and C) *E*. *coli* pBBRBB. Filter discs in each image are identical, (6 mm in diameter).

**Table 1:** Filter disc assay for mercury(II) chloride resistance in *E*. *coli*. Results are the average of three independent experiments with error represented as standard error of the mean.

Strain	Zone of Inhibition Diameter (mm)
*E*. *coli* pDU1358	16.5 ± 0.3
*E*. *coli* pBBRBB::*mer*	16.7 ± 0.7
*E*. *coli* pBBRBB	26.5 ± 0.3

To use engineered *E*. *coli* pBBRBB::*mer* cells in a filtration system, the cells must be fully encapsulated in silica microbeads to prevent release of biological material. Cells were mixed with a colloidal silica nanoparticle/PEG solution and then spiked with a hydrolyzed silicon TMOS solution. Transfer of this solution to aerated mineral oil enabled encapsulation of cells and resulted in the formation of smooth, spherical silica gel microbeads (Fig 2A). Microbead structures were chosen for encapsulation because they increase surface to volume ratio for bioremediation efforts and result in a biological-based filtration material that can be used in packed bed reactors. Measurement of 20 beads using a Hitachi scanning electron microscope indicated an average bead diameter of 210 ± 60 μm. Images also indicated that gel porosity was in the nanometer range, similar to previously characterized hyperporous beads generated using the same sol-gel methods, which limits mobility of encapsulated cells (Fig 2B) [23]. Because of the gel structure and limited space, cellular division is likely also inhibited. Despite limited space, use of PEG in silica bead formation has been shown to retain cell viability for at least three weeks following encapsulation [23].

**Fig 2:** Scanning Electron Microscopy images of encapsulation silica sol-gel microbeads containing *E*. *coli* pBBRBB::*mer*. A) Representative image depicting the smooth, spherical shape of silica microbeads following encapsulation in aerated mineral oil. Scale bar represents 200 μm B) Image of engineered *E*. *coli* pBBRBB::*mer* cells within encapsulation beads. Scale bar represents 5 μm.

Importantly, no cells were visualized on the surface of beads, and to image encapsulated cells, beads had to be crushed. Inside the gels, encapsulated cells appeared evenly dispersed within the gel matrix resulting in a highly porous material (Fig 2B). Encapsulated bacteria were found either as small clusters or as single cells throughout the gel. Encapsulated cells also retained normal cellular morphology and dimensions characteristic of *E*. *coli* (Fig 2B). Overall, resulting microbeads were within the diameter range and bacterial loading capacity shown in previous models to both maximize diffusion and maintain mechanical strength in flow-through systems [24].

To assess potential for degradation of methylmercury by *E*. *coli* pBBRBB::*mer*, both encapsulated and non-encapsulated cells were incubated in LB medium in the presence of 1 mg L^-1^ methylmercury chloride, which is a concentration 1000-fold greater than typically seen in contaminated environments and gold mining tailings ponds and thus a stringent test of our approach for methylmercury remediation [30, 31]. Samples were removed at various time points and analyzed for methylmercury concentration using a Tekran model 2700 Automated MethylMercury Analyzer with mercury detection by cold vapor atomic fluorescence spectrometry (CVAFS). Abiotic encapsulation beads and *E*. *coli* containing empty vector pBBRBB were included as negative controls.

*E*. *coli* pBBRBB::*mer* was efficient at remediation of methylmercury chloride prior to encapsulation. Non-encapsulated *E*. *coli* pBBRBB::*mer* was able to remediate greater than 99% of methylmercury chloride from solution after only 4 hours of incubation (Fig 3A). The rate constant for degradation of methylmercury chloride by *E*. *coli* pBBRBB::*mer* was 0.96 ± 0.07 hr-^1^ with a measured half-life for methylmercury chloride of 0.72 ± 0.07 hours (Fig 3A). Abiotic samples, as well as tubes containing non-encapsulated *E*. *coli* harboring an empty vector, showed slight decreases in the concentration of methylmercury after 24 hours (-0.16 ± 0.05 mg L^-1^ and -0.20 ± 0.05 mg L^-1^, respectively), and are likely due to photodecomposition of methylmercury [32] (Fig 3A). Taken together, these results indicate that the dramatically enhanced rate of methylmercury chloride degradation by *E*. *coli* pBBRBB::*mer* is due to Mer-mediated activity in engineered cells.

**Fig 3:** Degradation of methylmercury chloride by A) Non-encapsulated (open symbols) and B) Encapsulated (closed symbols) *E*. *coli* pBBRBB::*mer* (circles) and *E*. *coli* pBBRBB (squares). Degradation of methylmercury chloride in abiotic medium (open triangle) and sorption by abiotic beads (closed triangle) were included as controls. Data presented is for experiments performed at least in triplicate with error bars represented as SEM.

We next sought to determine if the rate of methylmercury degradation by encapsulated *E*. *coli* pBBRBB::*mer* was inhibited since encapsulation is likely to provide a diffusion barrier to degradation [33]. Methylmercury degradation rates were similar between non-encapsulated and encapsulated cells. The rate constant for degradation of methylmercury chloride by encapsulated *E*. *coli* pBBRBB::*mer* was 0.87 ± 0.04 hr^-1^ with a measured half-life for methylmercury chloride of 0.80 ± 0.04 hours (Fig 3B). Over 97% remediation of methylmercury chloride was achieved using encapsulated *E*. *coli* pBBRBB::*mer* after 4 hours of incubation (Fig 3B). These results suggest that encapsulation did not diminish the ability of *E*. *coli* pBBRBB::*mer* to degrade methylmercury.

Abiotic encapsulation beads were also incubated in the presence of methylmercury chloride to determine if the beads alone absorbed significant amounts of this compound. Only small concentrations of methylmercury chloride were absorbed by abiotic silica gel beads (-0.27 ± 0.06 mg L^-1^) as well as beads containing *E*. *coli* with the empty vector control (-0.20 ± 0.05 mg L^-1^) after 24 hours (Fig 3B). Absorption of methylmercury chloride by silica gel beads would aid in remediation efforts but would also hamper efforts to capture and potentially recycle elemental mercury using incorporated activated charcoal filters in scale-up packed bed reactors.

## Conclusion

Because mercury cannot be transformed into a non-toxic state, remediation efforts have focused on conversion of organic and ionic forms to the less toxic elemental form Hg(0). Ultimately, the goal of any mercury remediation strategy is to capture the elemental form, thereby enabling safe disposal and the potential to recycle materials. Encapsulation of bacterial cells containing the *mer* operon provide a possible answer to the challenges involved in mercury remediation since encapsulation enables use of engineered cells and the filtration material can be incorporated in flow-through systems.

By incorporating a subset of the *mer* operon in *E*. *coli* and encapsulating cells in silica beads, a remediation platform targeting both ionic and organic forms of mercury was developed. Performing encapsulation in aerated mineral oil resulted in the production of smooth, spherical beads (Fig 2) that could be incorporated into packed bed reactor treatment facilities. Encapsulated *E*. *coli* pBBRBB::*mer* performed similarly to non-encapsulated cells, and was able to remediate high methylmercury concentrations to below detection levels after approximately 4 hours (Fig 3). Encapsulation, by providing protection to the biocatalysts and overall mechanical structure, broadens possible engineering applications for the remediation of mercury. A possible scheme for methylmercury remediation based on this engineered, encapsulated system is outlined in Fig 4. Contaminated water is passed through the encapsulation beads where Mer-mediated activity catalyzes cleavage of the C-Hg bond of organic mercury species followed by reduction of Hg(II) to Hg(0) (mediated by MerA, encoded in pBBRBB::*mer*, but the activity was not tested here). A charcoal filter is incorporated downstream to capture mercury enabling recovery and proper disposal.

**Fig 4:** Process for utilizing silica-encapsulated *E*. *coli* pBBRBB::*mer* as a bioremediation catalyst in flow-through systems. *E*. *coli* containing pBBRBB::*mer* are encapsulated in silica beads using sol-gel technology and catalyze the cleavage of organic C-Hg bonds of mercury species and subsequent reduction of Hg(II) to Hg(0). Resulting Hg(0) is then captured downstream by an activated charcoal filter.

Mercury pollution is widespread, and its effects are not limited to areas near the source of pollution. Since mercury can travel thousands of miles through the atmosphere before being deposited back in the environment, it has become an issue of global concern. Remediation methods are needed that can target multiple arenas including industry, mining tailing ponds, and open bodies of water. This study provides a foundation for methods to encapsulate *mer*-containing bacteria in silica materials to offer a versatile option that can be tailored to various mercury-polluted sites. Further work in this area is being targeted at refactoring the *mer* operon to increase turnover rates, testing other genera such as encapsulated *Pseudomonas* species for the remediation of methylmercury, and determination of long-term cell escape rates from beads.
